# Stochastic Simulation of Typhoon in Northwest Pacific Basin Based on Machine Learning

**DOI:** 10.1155/2022/6760944

**Published:** 2022-02-17

**Authors:** Yong Fang, Yanhua Sun, Lu Zhang, Gengxin Chen, Mei Du, Yunxia Guo

**Affiliations:** ^1^College of Mathematics and Systems Science, Shandong University of Science and Technology, Qingdao 266590, China; ^2^State Key Laboratory of Tropical Oceanography, South China Sea Institute of Oceanology, Chinese Academy of Sciences, Guangzhou 510301, China; ^3^Department of Mathematical and Physics, Shijiazhuang Tiedao University, Shijiazhuang 050043, China

## Abstract

Typhoons have caused serious economic losses and casualties in coastal areas all over the world. The big size of the tropical cyclone sample by stochastic simulation can effectively evaluate the typhoon hazard risk, and the typhoon full-track model is the most popular model for typhoon stochastic simulation. Based on the advantages of machine learning in dealing with nonlinear problems, this study uses a backpropagation neural network (BPNN) to replace the regression model in the empirical track model, reestablishes the neural network model for track and intensity prediction in typhoon stochastic simulation, and constructs full‐track typhoon events of 1000 years for Northwest Pacific basin. The validation results indicate that the BPNN can improve the accuracy of typhoon track and intensity prediction.

## 1. Introduction

Typhoon is a strong disastrous weather system that occurs in the tropical ocean. It is commonly known as typhoon in the Northwest Pacific. The disasters such as strong wind, rainstorm, and huge waves caused by typhoon have led to serious social and economic losses and casualties in coastal areas. The southeast coastal region of China is one of the areas most seriously affected by typhoon in the world. From 1983 to 2008, the average economic losses caused by typhoons in China were about Chinese Yuan (CNY) 25 billion every year, and the loss showed an obvious growth trend [1, 2]. Taking the typhoon Meranti in 2016 as an example, it landed in Xiamen, Fujian Province, and it affected 3.04 million people in Fujian and Zhejiang provinces, with a direct economic loss of CNY 21.073 billion [3]. Therefore, accurate assessment of typhoon risk is very important for national disaster prevention and mitigation [4].

Typhoon risk analysis has strong statistical characteristics, and the results are often limited by the size and quality of samples. Therefore, the method of stochastic simulation to expand tropical cyclone (TC) samples for typhoon risk assessment has been developed internationally [5] and has gradually become an important research field of typhoon risk assessment. The general steps adopted for the typhoon risk analysis are as follows: First, the characteristics of tropical cyclones (TCs) are extracted from historical data for the construction of the typhoon stochastic model. Then, abundant virtual typhoons are simulated by the stochastic model to expand typhoon sample. Finally, the regional risk analysis is completed through the expanded samples. The two most widely accepted models for typhoon stochastic simulation are the circular subregion model and the empirical track model.

The circular subregion model is a traditional method of typhoon risk analysis. It was first implemented by Russell [6] for the estimation of typhoon wind speed on the Texas coast (US). Since then, many researchers [7-13] have done a lot of research work on the circular subregion model. They analyzed the typhoon risk combined with different typhoon wind field models for different research areas and achieved good results. Earlier in China, some researchers [14, 15] also used this model to analyze typhoon risk. Its basic steps are as follows: First, the historical typhoon events affecting a research site are extracted based on the circular subregion, and the typhoon key parameters are extracted, for example, central pressure difference, translation speed, storm heading, and annual occurrence rate. Next, the optimal probability distribution is fitted for each typhoon key parameter by probability distribution fitting. Third, the Monte Carlo method is used to sample from each probability distribution, generate massive key parameters of the virtual typhoon, and combine them to form virtual typhoon events. Fourth, the wind speed of the virtual typhoon is calculated by the typhoon wind field model, from which the typhoon maximum wind speed for one site can be obtained. Finally, the extreme wind speed of different return periods for a research site can be predicted by the extreme value distribution. The circular subregion model is generally applicable to small-scale areas with sufficient historical data of TCs and is not competent for typhoon risk analysis under future climate change [4].

The empirical track model is developed by Vickery et al. [16] which is the starting point for the development of the typhoon full-track model. They divided the whole Atlantic basin into nonoverlapping units and then build an empirical model of Hurricane track and intensity based on regression analysis from the historical TC data in each unit. There are many studies [17-27] for typhoon risk analysis based on the empirical track model. The setting of wind speed in the American building code is also based on this method [28]. The circular subregional model is suitable for analyzing the typhoon risk at a single site or in a small area because it depends on the assumption of typhoon climate uniformity in a small area. However, the empirical track model can produce a complete typhoon track. Therefore, it is suitable for analyzing the typhoon risk in a large area. Although there are many different modeling methods in the empirical track model, the basic idea is similar. First, the path is simulated in segments (generation model, movement model, intensity model, and extinction model) and then combined into a complete TC track. The physical meaning of each segment of the empirical track model is very clear. It can be said that the empirical track model is the most potential stochastic model to evaluate the risk of typhoon.

ANN is an algorithmic mathematical model for distributed parallel information processing by imitating the behavior characteristics of animal neural networks [29]. ANN has a strong learning ability and is good at simulating nonlinear system, which is suitable for predicting typhoon tracks and intensity. Among many training algorithms, the backpropagation neural network (BPNN) is still one of the most widely used models [30]. BPNN is based on the backpropagation learning theory of a multilayer feedforward neural network. It has the characteristics of simple structure, stable working state, and easy implementation. In recent years, many international researchers have applied artificial neural network (ANN) based on massive data to predict the typhoon track or intensity [30-34]. Wang et al. [30] used BPNN for typhoon track prediction in the Northwest Pacific basin. They normalized the TC data and input it into BPNN, breaking the limitation of long-term manual construction of prediction factors. Baik [35] used BPNN to forecast typhoon intensity and compared it with the regression method. The results show that the prediction error of BPNN is less than that of the regression method, which indicates the prospect of BPNN in typhoon intensity prediction. Zhou et al. [36] predicted the typhoon track with the improved BP model. The results showed that the coincidence rate between the storm heading predicted by ANN and the actual TC path was 97%. Shao et al. [37] used the BP model to predict the typhoon tracks along the Chinese coast and compared the prediction results with those of the climatology and persistence (CLIPER) model. The results show that the forecast accuracy of the BP model is higher than that of the CLIPER model.

The traditional empirical track model uses a statistical regression method to predict the typhoon track and intensity, which could not escape some forecast errors. ANN method has better adaptive learning and nonlinear mapping ability. It is more suitable to deal with nonlinear problems with complicated physical mechanism, causality, or reasoning rules. Therefore, this study intends to use BPNN to reestablish the prediction model of typhoon track and intensity in typhoon stochastic simulation, to improve the accuracy of typhoon track and intensity prediction, and then to improve the accuracy of typhoon risk analysis.

## 2. Methods

### 2.1. Empirical Track Model

The storm empirical track model was developed by Vickery et al. [16], which describes the changes of translation speed *c*, storm heading *θ*, and intensity *I* of typhoon at two adjacent moments. The model is described as follows:

(1a) $$\begin{array}{c} \Delta \;\ln\;c=a_{1}+a_{2}\psi +a_{3}\lambda +a_{4}\ln\;c_{i}+a_{5}\theta_{i}+\varepsilon_{c}, \end{array}$$

(1b) $$\begin{array}{c} \Delta \theta =b_{1}+b_{2}\psi +b_{3}\lambda +b_{4}c_{i}+b_{5}\theta_{i}+b_{6}\theta_{i-1}+\varepsilon_{\theta }, \end{array}$$

(1c) $$\begin{array}{c} \ln\left(I_{i+1}\right)=d_{1}+d_{2}\ln\left(I_{i}\right)+d_{3}\ln\left(I_{i-1}\right)+d_{4}\ln\left(I_{i-2}\right)+d_{5}Ts_{i}+d_{6}\left(Ts_{i+1}-Ts_{i}\right)+\varepsilon_{I}. \end{array}$$

where *a*_1_, *a*_2_, etc. are constants; Ψ represents the latitude (°) of typhoon center; *λ* represents the longitude (°) of typhoon center; *c* is the Hurricane translation speed (m/s); *θ* is the storm heading (°); *I* is the Hurricane relative intensity; *i*-1, *i*, and *i*+1 represent different time steps; the time interval between *i* + 1 and *i* is 6 h; Δln*c* = ln*c*_i+1_ − ln*c*_i_ and Δ*θ* = *θ*_*i*+1_ − *θ*_*i*_; *T*_S*i*_ is the monthly averaged sea surface temperature (SST, °K); and *ε*_c_, *ε*_*θ*_, and *ε*_*I*_ are random error terms with zero mean.

The concept of typhoon relative intensity was proposed by Darling [38] based on the principle of the Carnot cycle heat engine. The relative intensity is expressed as follows:

(2) $$\begin{array}{c} I=\left(p_{da}-p_{c}+e_{s}\right)/\left(p_{da}-p_{dc}\right), \end{array}$$

where *p*_da_ is the ambient pressure (hPa); *p*_dc_ is the minimum sustainable surface value of central dry partial pressure (hPa); *p*_c_ is the typhoon central pressure (hPa); and *e*_*s*_ is the saturation vapor pressure.

Vickery et al. [16] divided the entire Atlantic basin into a 5° × 5° grid. Based on the historical Hurricane data of each grid, the coefficients *a*_1_, *a*_2_, etc. of the regression model are fitted. In addition, they distinguished the easterly and westerly headed storms and obtained two different sets of model coefficients. For some grid cells with too few historical Hurricane data, the fitted regression model is not reliable, so the reliable regression model of a nearby grid cell is used instead.

The original empirical track model has many coefficients that need to be estimated for each grid cell. Li and Hong [22] simplified the storm track modeling of Vickery et al. [16] based on the geographically weighted regression method implemented in ArcGIS [39] and verified the effectiveness of the simplified model. The simplified track modeling is defined as follows:

(3a) $$\begin{array}{c} \Delta \;\ln\;c=a_{1}+a_{2}\ln\;c_{i}+a_{3}\theta_{i}+\varepsilon_{c}, \end{array}$$

(3b) $$\begin{array}{c} \Delta \theta =b_{1}+b_{2}c_{i}+b_{3}\theta_{i}+\varepsilon_{\theta }, \end{array}$$

(3c) $$\begin{array}{c} \ln\left(I_{i+1}\right)=d_{1}+d_{2}\ln\left(I_{i}\right)+d_{3}Ts_{i}+d_{4}\left(Ts_{i+1}-Ts_{i}\right)+\varepsilon_{I}. \end{array}$$

### 2.2. Backpropagation Neural Network (BPNN)

Artificial neural networks (ANNs) can model any input and corresponding output without considering the interaction mechanism between them [40]. It processes information by adjusting the interconnected relationship among a large number of internal nodes (or neurons) [29]. Readers can refer to [29, 41] for more details about ANN.

This paper adopts BP neural network, which is widely used in the artificial neural network, including input layer, hidden layer, and output layer (Figure 1). BPNN derives from the fact that in the neutral network, information data are passed feedforward from the input layer to the output layer, and then, the errors are propagated back. BP algorithm is actually a generalized form of the least mean square algorithm [30, 42]. It uses gradient steepest descent technology to recursively solve the weight of the network and the threshold of each node according to the criterion of minimizing the mean square error of the actual output and expected output of the network. In the feedforward process, the information data are inputted to the nodes of the input layer and then are transmitted to the output layer after processing by the hidden layer (see Figure 1). If the actual output of the output layer does not match the target output, it turns to the backpropagation stage of the error (Figure 1). It is always difficult to determine the hidden layer number in ANN. Schroeder et al. [43] suggested that one hidden layer is sufficient for most purposes. Thus, only one hidden layer was used in this study for simplicity.

We selected the most used “maximum squared error” (MSE) as the performance function of the BP network training, which can evaluate the simulating performance of the network.

(4) $$\begin{array}{c} MSE=\frac{1}{2m}\sum_{k=1}^{m}\sum_{t=1}^{q}{\left(y_{t}^{k}-c_{t}^{k}\right)}^{2}, \end{array}$$

where *y*_*t*_ is the target output and *c*_*t*_ is the network output. A set of the input vector and corresponding target output vector constitutes a training pattern of the network, *m* represents the total number of training patterns, and *q* is the number of neurons in output layer. The error at the output layer is backpropagated and is allocated to all nodes of each layer as the basis for adjusting the weight of each node. The interconnection weights and biases are iteratively adjusted in the feedforward process and error back propagation. The iteration process continues, until a specified convergence is reached or until a predetermined number of learning times [44].

## 3. Materials

The historical typhoon dataset used for this study comes from the Yearbook of Tropical Cyclone provided by the China Meteorological Administration (CMA) (1949–2019, from tcdata.typhoon.org.cn). The data were first released by the China Central Meteorological Observatory (CCMB) (from 1949 to 1982) and then released by the China National Meteorological Administration (CNMB) (from 1983 to 1992). Since then, it has been maintained and updated by CMA. The database records the relevant information of all tropical cyclones passing through the Northwest Pacific and the South China Sea since 1949. It contains the location and intensity information of typhoons at a time interval of 6 h, including the name and number of typhoons, typhoon center position (longitude and latitude), central pressure, and 2-min mean maximum sustained wind speed near the center (MSW, m/s).

Due to the use of different anemometers, the data from 1949 to 1970 are relatively large compared with the later data. Therefore, before using the typhoon data provided by the CMA, this paper corrected the data before 1970 based on the correction method of Li et al. [45]. And the tropical depressions and denatured typhoons were eliminated from the historical dataset [46].

The SST data used in this study in the typhoon intensity model are from the moderate resolution imaging spectroradiometer (MODIS) ocean products [47]. MODIS is a key instrument aboard the Terra and Aqua satellites, which are used to measure global climate change.

## 4. BP Network and Training

### 4.1. Selecting of Input Data and Target Data

First, we divided the Northwest Pacific basin into 5° × 5° grid, and the grid number is shown in Figure 2(a). Then, the prediction models of typhoon translation speed, storm heading, and intensity for each grid were established based on the historical typhoon data in each grid. When the number of historical typhoons in a grid is less than 15, the coefficients or the prediction models were replaced with those of the nearest grid cell. There are many factors affecting the typhoon track and intensity, for example, typhoon position, translation speed, and storm heading of the typhoon at the former 6-hour time, and air-sea background environment of the typhoon. Referring to previous research studies [16, 22], for the prediction model of typhoon translation speed, we selected the typhoon translation speed, storm heading, and the typhoon position (longitude and latitude) at the former 6-hour time, that is, *c*_*i*_, *θ*_*i*_, *ψ*, and *λ*, as the input data, and the translation speed at the next adjacent time, that is, *c*_*i*+1_, as the output data. For the prediction model of storm heading, the input data are the same as that of the typhoon translation speed model, and the output is the storm heading of the next adjacent time, that is,*θ*_*i*+1_. When selecting the relative intensity *I* and sea surface temperature *T*_*s*_ as the input data for the typhoon intensity model, we found the predicted typhoon intensity was easy to jump. This is mainly because the calculation formula of relative intensity is too complex, and the neural network is prone to overfitting in the grid cells with less historical typhoon data. Therefore, we directly selected the typhoon central pressure at the former 6-hour and 12-hour time and the SST at the former 6-hour time, that is, *p*_*i*_, *p*_*i*-1_, and *Ts*_*i*_, as the input data, and the typhoon central pressure at the next adjacent time, that is, *p*_*i*+1_, as the output data.

### 4.2. Establishment of the BP Model

A training pattern for the prediction model of typhoon translation speed is *c*_*i*_, *θ*_*i*_, *ψ*, *λ*, and *c*_*i*+1_. That for the prediction model of storm heading is *c*_*i*_, *θ*_*i*_, *ψ*, *λ*, and *θ*_*i*+1_. *P*_*i*_, *p*_*i*-1_, *Ts*_*i*_, and *p*_*i*+1_ form the training pattern for the typhoon intensity model. Based on the statistical results of historical typhoon data from CMA data, the number of training pattern for easterly and westerly headed storms in each grid is shown in Figures 2(b) and 2(c).

There are many parameters to be determined in a BPNN model, for example, the number of nodes in each layer of neural network, the activation function, and the training function.

The node number in input (output) layer depends on the dimension of the input (output) vector. Based on the research results of Vickery et al. [16] and Li et al. [22], present study built different neutral networks for each typhoon translation speed model, storm heading model, and intensity model considering different training patterns of input and corresponding output vectors, as shown in Table 1.

There is still no better method to determine the number of nodes in the hidden layer in advance. Too few nodes will make the network performance poor, and too many nodes will prolong the training time and prone to overfitting. Therefore, the node number is usually gradually increased or reduced in the training process, until the required accuracy is achieved. After debugging by trial and error method, the node number of the hidden layer is determined to be 10 (only one hidden layer). When the node number of the hidden layer is 10, for most grid cells, the correlation coefficient between neural network prediction results and actual results is the largest, and the root mean square error is the smallest.

### 4.3. Evaluation Index

In order to evaluate the prediction results under different neural network models, the correlation coefficient (*R*) and root mean square error (*RMSE*) between the predicted and target results were adopted in this study. The calculation formulas are as follows:

(5) R=∑k=1nyk−yk¯y^k−y^k¯∑k=1nyk−yk¯2∑k=1ny^k−y^k¯2,

(6) $$\begin{array}{c} RMSE=\sqrt{\frac{\sum_{k=1}^{n}\left(y_{k}-{\hat{y}}_{k}\right)}{N}}. \end{array}$$

where *y*_*k*_ denotes the predicted results of the network and ${\hat{y}}_{k}$ represents the actual observed results. $\bar{y_{k}}$ is the average value of predicted results, $\bar{y_{\text{k}}}=1/n\sum_{k=1}^{n}y_{k}$. $\bar{{\hat{y}}_{k}}$ indicates the average value of the actual observed results, $\bar{{\hat{y}}_{k}}=1/n\sum_{k=1}^{n}{\hat{y}}_{k}$. The correlation coefficient is used to evaluate the strength of the correlation between the predicted and the observed results. The closer the absolute value |*R*| is to 1, the stronger the correlation is. The *RMSE* represents the error between the values of prediction and actual observation. The smaller the error is, the more accurate the predicted value is.

## 5. Training Results and Validation

### 5.1. Results of Training

Figure 3 shows the comparison of correlation coefficients between the different neural network models for each grid cell.  Figure 3(a) shows the comparison results of different typhoon translation speed models, Figure 3(b) shows those of different storm heading models, and Figure 3(c) shows those of different central pressure models. The statistical results of *R* and *RMSE* for each typhoon prediction model are shown in Table 2.

We can see from Table 2 that, for the prediction model of the typhoon translation speed, the average correlation coefficient from ANNa2 is the highest, and the average *RMSE* is the smallest. Therefore, ANNa2 is adopted as the optimal prediction model of typhoon translation speed. For the prediction model of storm heading, the prediction results of ANNb2 are better than those of ANNb1. Therefore, ANNb2 is selected as the optimal prediction model of storm heading. For the prediction model of typhoon central pressure, the prediction results of the ANNc1 are better than those of ANNc2. Therefore, ANNc1 is chosen as the optimal prediction model of typhoon central pressure.

In order to reflect the advantage of the neural network prediction model, we compared the correlation coefficient and *RMSE* from the neural network prediction model with the results of the traditional regression model [22]. The optimal prediction models of the neural network for typhoon translation speed, storm heading, and central pressure are ANNa2, ANNb2, and ANNc1, and the corresponding regression models are formulas 1(a), formula 3(b), and the following formula, respectively:

(7) $$\begin{array}{c} \Delta p=d_{1}+d_{2}p_{i}+d_{3}p_{i-1}+d_{4}Ts_{i}+\varepsilon_{p}. \end{array}$$

Figure 4 shows the differences of correlation coefficient (or *RMSE*) of typhoon translation speed predicted by the BP model (ANNa2) and regression model (formula 1(a)) for each grid cell. The comparison of the prediction results for easterly headed storms is shown in Figures 4(a) and 4(b), and that for westerly headed storms is shown in Figures 4(c) and 4(d). It can be seen from Figures 4(a) and 4(c) that, for each grid cell, the correlation of typhoon translation speed between the results of the BP model and the observed values is better than the result of the regression model for both easterly and westerly headed storms. Figures 4(b) and 4(d) show that, for each grid cell, the *RMSE* of typhoon translation speed between the BP model and the observed values is smaller than that of the regression model for both easterly and westerly headed storms. All the above indicates that, for the prediction of typhoon translation speed, the prediction results of the BP model are better than those of the regression model.

Figure 5 shows the differences of correlation coefficient (or *RMSE*) of storm heading predicted by the BP model (ANNb2) and regression model (formula (3b)) for each grid cell. The comparison of the prediction results for easterly headed storms is shown in Figures 5(a) and 5(b), and that for westerly headed storms is shown in Figures 5(c) and 5(d). It can be seen from Figures 5(a) and 5(c) that, for each grid cell, the correlation of storm heading between the results of the BP model and the observed values is better than the result of the regression model for both easterly and westerly headed storms. Figures 5(b) and 5(d) show that, for each grid cell, the *RMSE* of storm heading between the BP model and the observed values is smaller than that of the regression model for both easterly and westerly headed storms. All the above indicates that, for the prediction of storm heading, the prediction results of the BP model are better than those of the regression model.

Figure 6 shows the differences of correlation coefficient (Figure 6(a)) and *RMSE* (Figure 6(b)) of typhoon central pressure predicted by the BP model (ANNc1) and regression model (formula (7)) for each grid cell. It can be seen from Figure 6(a) that, for most grid cells, the correlation of typhoon central pressure between the results of the BP model and the observed values is better than the result of the regression model. Figure 6(b) shows that, for most grid cells, the *RMSE* of typhoon central pressure between the BP model and the observed values is smaller than that of the regression model. All the above indicates that, for the prediction of typhoon central pressure, the prediction results of the BP model are better than those of the regression model.

### 5.2. Validation of BP Models

The process of constructing a virtual typhoon is to first divide the Northwest Pacific basin into a 5° × 5° grid and then build a neural network prediction model (or statistical regression prediction model) for the typhoon translation speed, storm heading, and intensity (central pressure) based on the historical typhoon data of each grid. Third, based on the distribution of the starting points of historical typhoons, the starting points of virtual typhoons are randomly selected to initialize the typhoon track. Fourth, the typhoon track and intensity prediction model of the grid where the typhoon is located are used to predict the typhoon position and intensity at the next time. Finally, the complete typhoon track can be obtained by repeating the fourth step.

Based on the above method of constructing a virtual typhoon, we constructed a virtual typhoon dataset of 1000 years for Northwest Pacific basin based on the BP model, including 32693 virtual typhoon events.  Figure 7 shows the comparison of the virtual and observed typhoon tracks.  Figure 7(a) shows all the observed typhoon tracks (2384 typhoon events in total) during 1949–2019.  Figure 7(b) shows the 71-year typhoon tracks randomly extracted from the virtual typhoon dataset constructed by the BP model. The comparison results indicate that the distribution of virtual typhoon tracks is almost consistent with that of observed typhoon tracks. However, since the termination of the virtual typhoons is artificially set to 1002 for typhoon central pressure, it is relatively uniform compared with the observed typhoons at the end of the typhoon track.

Taking the super typhoon Lekima, which landed in China in 2019, as an example, we used the constructed BP neural network model to predict 12 typhoon tracks that have the same initial state as Lekima, and the predicted and observed typhoon paths are shown in Figure 8. It can be seen from Figure 8 that the moving trend of most virtual typhoon tracks is consistent with the observed typhoon track, and half of the typhoon tracks are very close to the observed typhoon track, indicating that the virtual typhoon tracks constructed by the BP neural network model are really credible.

To further validate the reliability of the virtual typhoon dataset constructed based on the BP model, we first selected 46 research stations at a space interval of 100 km along the east coast of China, as shown in Figure 9. Then, we extracted the typhoon events that affect each station from the virtual typhoon dataset and the historical typhoon dataset, respectively. The extraction method is to delimit a circular subregion with a radius of 250 km with each station as the center of the circle. When the typhoon passes through the circular subregion, it will be regarded as a typhoon event affecting the station. Li and Hong [22, 25] and Vickery et al. [48] also used 250 km as the radius of the circular subregion. Third, the key parameters of typhoon events are counted when they are closest to each station, including typhoon annual occurrence rate, translation speed, and storm heading, and furthermore, the mean or standard deviations of these parameters are counted. The parameter of typhoon central pressure was defined as the minimum value of typhoon central pressure within the 250 km subregion. In addition, we also constructed a virtual typhoon dataset of 1000 years for the Northwest Pacific basin based on the regression model and compared its statistical results with those of the BP model.

Figure 10 compares the means and standard deviations of key parameters of typhoons simulated by the BP model (Figures 10(a) and 10(c)) or regression model (Figures 10(b) and 10(d)) and those of observed typhoons for each research station along China's coastline. Overall, the statistical characteristics of virtual typhoons constructed by the BP model or regression model are consistent with those of observed typhoons. For annual occurrence rate, the statistical results from the BP model are in good agreement with the observed results, while the statistical results from the regression model are different from the observed results along the coast of Zhejiang, Fujian, and Guangdong Province. For the central pressure difference of typhoon, the statistical results from the BP model are in good agreement with the observed results, while the statistical results from the regression model are slightly different from the observed results along the coast of Fujian and Guangdong Province. For typhoon translation speed, the statistical results from two different models do not match the observed results along the coast of Liaoning, Hebei, and Shandong Province, while the statistical results from the regression model are worse along the coast of Hebei and Northern Shandong Province. For storm heading, the statistical results from two different models match well with the observed results. We can conclude that the virtual typhoons constructed by the BP model and regression model reproduce the statistical characteristics of coastal typhoons in China, and the BP model works better.

## 6. Conclusion

Artificial neural network has better self-adapting, self-learning, and nonlinearity mapping capability, which is more suitable for dealing with complex nonlinear problems. This paper used BP neural network to replace the regression model in the original typhoon empirical track model and reestablished prediction models of typhoon track and intensity in typhoon stochastic simulation. For the prediction models of typhoon translation speed, storm heading, and typhoon central pressure, different input and output factors were used to establish different BP models, and the optimal model was selected through model evaluation. Based on the optimal models of typhoon translation speed, storm heading, and typhoon central pressure, this paper constructs virtual typhoon events of 1000 years for Northwest Pacific basin. The validation results indicate that the BPNN can improve the prediction accuracy of typhoon track and intensity.

## Figures and Tables

**Figure 1:** Schematic diagram of a three-layer neural network.

**Figure 2:** (a) The number of grid cell of 5° × 5° in Northwest Pacific Ocean and the number of training pattern in each grid from (b) easterly and (c) westerly headed storms.

**Figure 3:** Comparison of correlation coefficients (*Rs*) between the different neural network models for each grid cell. Taking the westerly headed storms as examples, the results for the easterly headed storms are similar: (a) comparison of *Rs* between the different neural network models for typhoon translation speed, (b) comparison of *Rs* between the different neural network models for the storm heading, and (c) comparison of *Rs* between the different neural network models for typhoon central pressure.

**Figure 4:** The differences of correlation coefficient and RMSE of typhoon translation speed predicted by the BP model (ANNa2) and regression model (formula 1(a)) for each grid cell. The differences of correlation coefficients from the BP model and the regression model for (a) easterly and (c) westerly headed storms. The differences of RMSE from the BP model and regression model for (b) easterly and (d) westerly headed storms.

**Figure 5:** The differences of correlation coefficient and *RMSE* of storm heading predicted by the BP model (ANNb2) and regression model (formula 3(b)) for each grid cell. The differences of correlation coefficients from the BP model and the regression model for (a) easterly and (c) westerly headed storms. The differences of *RMSE* from the BP model and regression model for (b) easterly and (d) westerly headed storms.

**Figure 6:** The differences of (a) correlation coefficient and (b) *RMSE* of typhoon central pressure predicted by the BP model (ANNc1) and regression model (formula 14) for each grid cell.

**Figure 7:** (a) The observed typhoon tracks during 1949–2019. (b) The 71-year typhoon tracks were randomly extracted from the virtual typhoon dataset constructed by the BP model.

**Figure 8:** The observed typhoon track of Lekima (2019) and the virtual typhoon tracks constructed by the BP model, which have the same initial state as Lekima.

**Figure 9:** Distribution of research stations (blue box) along the China coastline used for validation.

**Figure 10:** Comparisons of the means and standard deviations of key parameters from virtual and observed typhoons at 46 coastal stations in China. (a) The results of the BP model, and (b) the results of the regression model.

**Table 1:** Setting of input and output layers in the neural network.

Prediction model	Name of the neural network	Input data	Node number of the input layer	Output data	Node number of the output layer
Typhoon translation speed model	ANNa1	*c*_*i*_, *θ*_*i*_, *ψ*, and *λ*	4	*c*_*i*+1_-*c*_*i*_	1
	ANNa2	ln*c*_*i*_, *θ*_*i*_, *ψ*, and *λ*	4	ln*c*_*i*+1_-ln*c*_*i*_	1
	ANNa3	ln*c*_*i*_, *θ*_*i*_	2	ln*c*_*i*+1_-ln*c*_*i*_	1

Storm heading model	ANNb1	*c*_*i*_, *θ*_*i*_, *θ*_*i*-1_, *ψ*, and *λ*	5	*θ*_*i*+1_-*θ*_*i*_	1
	ANNb2	*c*_*i*_, *θ*_*i*_	2	*θ*_*i*+1_-*θ*_*i*_	1

Typhoon intensity model	ANNc1	*p*_*i*_, *p*_*i*-1_, and *Ts*_*i*_	3	*p*_*i*+1_-*p*_*i*_	1
	ANNc2	*p*_*i*_, *Ts*_*i*_	2	*p*_*i*+1_-*p*_*i*_	1

**Table 2:** Statistical results of the correlation coefficient and the root mean square error for each typhoon prediction model.

Statistics	ANNa1	ANNa2	ANNa3	ANNa1	ANNa2	ANNa3
	-East	-East	-East	-West	-West	-West
Mean of *R*	0.53	**0.77**	0.68	0.50	**0.68**	0.62
Mean of *RMSE*	4.67	**0.13**	0.17	3.74	**0.15**	0.18

Statistics	ANNb1	ANNb2	ANNb1	ANNb2	ANNc1	ANNc2
	-east	-east	-West	-West		
Mean of *R*	0.47	**0.60**	0.41	**0.49**	**0.64**	0.52
Mean of *RMSE*	17.54	**15.58**	13.29	**12.66**	**2.09**	2.27

## Data Availability

The data in this study are from the CMA-STI (China Meteorological Administration and Shanghai Typhoon Institute) Best Track Dataset for Tropical Cyclones over the Western North Pacific (http://tcdata.typhoon.org.cn).
